The article "Atom Search Optimization with the Deep Transfer Learning-Driven Esophageal Cancer Classification Model" was retracted in 2023. Reasons: signs of a paper mill; suspected computer-generated content; unreliable results or conclusions; concerns about the data.

# Atom Search Optimization with the Deep Transfer Learning-Driven Esophageal Cancer Classification Model

**DOI:** 10.1155/2022/4629178

**Published:** 2022-09-16

**Authors:** Nawaf R. Alharbe, Raafat M. Munshi, Manal M. Khayyat, Mashael M. Khayyat, Saadia Hassan Abdalaha Hamza, Abeer A. Aljohani

**Affiliations:** ^1^Applied College, Taibah University, Medina, Saudi Arabia; ^2^Department of Medical Laboratory Technology (MLT), Faculty of Applied Medical Sciences, King Abdulaziz University, Rabigh, Saudi Arabia; ^3^Department of Information Systems, College of Computers and Information Systems, Umm Al-Qura University, Makkah, Saudi Arabia; ^4^Department of Information Systems and Technology, Faculty of Computer Science and Engineering, University of Jeddah, Jeddah, Saudi Arabia; ^5^Department of Computer Science College of Science and Humanities in Al-Sulail, Prince Sattam Bin Abdulaziz University, Saudi Arabia

## Abstract

Esophageal cancer (EC) is a commonly occurring malignant tumor that significantly affects human health. Earlier recognition and classification of EC or premalignant lesions can result in highly effective targeted intervention. Accurate detection and classification of distinct stages of EC provide effective precision therapy planning and improve the 5-year survival rate. Automated recognition of EC can aid physicians in improving diagnostic performance and accuracy. However, the classification of EC is challenging due to identical endoscopic features, like mucosal erosion, hyperemia, and roughness. The recent developments of deep learning (DL) and computer-aided diagnosis (CAD) models have been useful for designing accurate EC classification models. In this aspect, this study develops an atom search optimization with a deep transfer learning-driven EC classification (ASODTL-ECC) model. The presented ASODTL-ECC model mainly examines the medical images for the existence of EC in a timely and accurate manner. To do so, the presented ASODTL-ECC model employs Gaussian filtering (GF) as a preprocessing stage to enhance image quality. In addition, the deep convolution neural network- (DCNN-) based residual network (ResNet) model is applied as a feature extraction approach. Besides, ASO with an extreme learning machine (ELM) model is utilized for identifying the presence of EC, showing the novelty of the work. The performance of the ASODTL-ECC model is assessed and compared with existing models under several medical images. The experimental results pointed out the improved performance of the ASODTL-ECC model over recent approaches.

## 1. Introduction

Esophageal cancer (EC) affects 3000 women and 13,480 men yearly in the US. Amongst males, it is considered the 7th leading cause of death globally. The occurrence rate was slowly increasing in males in Japan. Even though progressions were made in surgery and perioperative management policies, long-term diagnosis of esophageal cancer, specifically in advanced levels, will be lower; the five-year endurance rate of patients with phase IV EC is nearly 20% in Japan [1]. In several cases, the indication of common digestive signs associated with EC, like difficulty in swallowing and heartburn, happens in developed phases. Moreover, esophagectomy, the common medication for phase II or III EC, is a very aggressive process accompanying higher rates of postoperative complexities like anastomotic leakage, pneumonia, and recurrent nerve palsy [2]. Postoperative complexities are linked with perioperative death, along with a rise in medical expenses, longer hospitalization, and delay of postoperative therapy [3]. At the same time, tumors identified in prior levels could be diagnosed with fewer aggressive processes like an endoscopic resection. Also, prior identification is linked with enhanced patient's diagnosis [4]. Thus, the initial identification of EC is vital.

The article "Atom Search Optimization with the Deep Transfer Learning-Driven Esophageal Cancer Classification Model" was retracted in 2023. Reasons: signs of a paper mill; suspected computer-generated content; unreliable results or conclusions; concerns about the data.

Precise staging, medication planning, and prognostication in EC patients are very important. Recently, researchers have looked at original applications like radionics by employing noninvasive imaging methodologies for improvising the patient's path [5]. Formerly concealed data could be discovered amongst distinct imaging modalities that can imitate the pathogenesis of EC. Positron emission tomography (PET), computed tomography (CT), generally blended with CT (PET-CT), ultrasonography endoscopic (EUS), and magnetic resonance imaging (MRI) are generally utilized for follow-up and staging [6]. CT and PET are the two modalities majorly utilized for EC patients. However, its capabilities to discover minor-sized lesions were confined, which disturbs the specificity and sensitivity of disease recognition [7]. Currently, AI is especially deep learning (DL) and has resulted in the expansion of image analysis, a method used for several intentions involving the categorization of skin cancer and identification of diabetic retinopathy in fundus images, pulmonary lesions in CT images, and upper gastrointestinal cancer in the endoscopic image [8–10]. A convolutional neural network (CNN) permits computational copies made up of numerous processing layers for learning illustrations of image data and has manifold stages of abstraction [11, 12]. It may also find new kinds of paradigm over subtle common radiographic characteristics that may aid us in preventing misunderstandings in recognition of cancerous lesions and helps in reducing the workload on radiotherapists.

The article "Atom Search Optimization with the Deep Transfer Learning-Driven Esophageal Cancer Classification Model" was retracted in 2023. Reasons: signs of a paper mill; suspected computer-generated content; unreliable results or conclusions; concerns about the data.

This study develops an atom search optimization with a deep transfer learning-driven EC classification (ASODTL-ECC) model. The presented ASODTL-ECC model employs Gaussian filtering (GF) as a preprocessing stage to enhance image quality. In addition, the deep convolution neural network- (DCNN-) based residual network (ResNet) technique was executed as a feature extraction approach. Besides, ASO with an extreme learning machine (ELM) model is utilized to identify the presence of EC. The performance of the ASODTL-ECC model is assessed and compared with existing models under several medical images.

The rest of the article is organized as follows: Section 2 reviews the recently developed EC classification models.  Section 3 offers a brief discussion of the proposed model and Section 4 provides experimental validation. At last, Section 5 concludes the study.

## 2. Prior EC Detection and Classification Models

Guo et al. [13] proposed a computer-assisted diagnosis (CAD) system for real-time automatic diagnoses of precancerous lesions and earlier esophageal squamous cell carcinomas (ESCCs) for assisting the diagnoses of esophageal lesions. The yellow color specifies a higher chance of cancerous tumor, and the blue color indicates a noncancerous lesion on the probability heatmap. Mubarak [14] conducted research on the classification of Barrett's esophagus (BE) and esophagitis with deep CNN (DCNN). CNNs with powerful feature extractors allow the optimum prognosis of Barrett's esophagus, esophagitis, and precancerous phase. The transfer learning technique using CNN extracts feature for the automatic classification of esophagitis and Barrett's esophagus.

Wang et al. [15] developed various paradigms based on the Kohonen network clustering technique and the kernel extreme learning machine (KELM), which aims at classifying the tested population into five categories and offer improved performance by using machine learning technique. The Taylor formula was utilized for expanding the concept to analyze the effect of activation function on the KELM modeling effect. RBF was carefully chosen as the different activation functions of the KELM. Lastly, the adoptive mutation sparrow search approach (AMSSA) was utilized to optimize the model parameter. Chen et al. [16] presented an EC diagnosis with the DL method for improving the detection accuracy and reducing the work intensity of doctors. In this article, the Fast-RCNN EC diagnosis presents the online hard example mining (OHEM) method.

Yeh et al. [17] aim to predict the existence of LVI and PNI in esophageal squamous cell carcinoma with a PET imaging dataset by training a 3DCNN. Initially, we constructed a 3DCNN dependent upon ResNet for classifying the scan into esophageal or lung cancers. Next, we gathered the PET scan of 278 patients enduring esophagectomy to predict and classify the existence of PNI or LVI. Cho et al. [18] used a CNN method, a DL technique, to categorize EC automatically and differentiate them from premalignant lesions. The presented CNN architecture comprises two subnetworks (O-stream and P-stream). The novel image was utilized as the input of the O-stream for extracting the global and color features, and the preprocessed esophageal image was utilized as the input of the P-stream for extracting the detail and texture features. Different studies have been conducted in the literature that focused on detecting EC. At the same time, the existing models do not focus on the hyperparameter selection process, which mainly influences the classification model's performance. Particularly, hyperparameters such as epoch count, batch size, and learning rate selection are essential to attain an effectual outcome. Since the trial and error method for parameter tuning is a tedious and erroneous process, metaheuristic algorithms can be applied. Therefore, in this work, we employ the ASO algorithm for the parameter selection of the ELM model.

The article "Atom Search Optimization with the Deep Transfer Learning-Driven Esophageal Cancer Classification Model" was retracted in 2023. Reasons: signs of a paper mill; suspected computer-generated content; unreliable results or conclusions; concerns about the data.

## 3. Materials and Methods

In this study, a novel ASODTL-ECC model was established to investigate the medical images for the existence of EC in a timely and accurate manner. The presented ASODTL-ECC model encompasses various subprocesses, namely, GF-based noise elimination, ResNet101-based feature extraction, ELM classification, and ASO-based parameter tuning. The use of the ASO algorithm assists in improving the identification of the presence of EC.  Figure 1 depicts the block diagram of the ASODTL-ECC approach. Initially, the medical images are preprocessed to remove the noise present in it. Then, they are fed into the ResNet101 model to generate feature vectors. Finally, the ASO with ELM model is utilized for the EC classification process.

### 3.1. Image Preprocessing

At the primary level, the presented ASODTL-ECC model exploited the GF technique as a preprocessing stage to enhance the image quality. GF approach minimizes pixels' variations through weight average for image smoothing from several applications. But, this low pass filter does not conserve particulars of the image, i.e., textures and edges. The linear translation variant functions *f* and next explains the aforementioned filter procedure as follows [19]:

(1) $$\begin{array}{c} f\left(p\right)=\underset{q}{\sum }K_{p,q}\left(Q\right)P_{q}\text{,} \end{array}$$

where *K*_*p*,*q*_ indicates every pixel *q* centered at pixel *p* from the filtering kernel *K*, and *Q* and *P* are input and guidance images, correspondingly. For instance, the kernel of the bilateral filter (BF) defined by (1) was expressed:

(2) $$\begin{array}{c} K_{p,q}\left(Q\right)=\frac{1}{n}\exp\left(-\frac{{\left\|p-q\right\|}^{2}}{\sigma_{s}^{2}}\right)\exp\left(-\frac{{\left\|P_{p}-Q_{q}\right\|}^{2}}{\sigma_{r}^{2}}\right)\text{,} \end{array}$$

where *n* refers the normalized factor and *σ*_*s*_ and *σ*_*r*_ denote the window size of neighborhood expansions and the alteration of edge amplitude intensities, respectively. The exponential distribution function was usually utilized in (2) for calculating the effect of distinct spatial distances by exp(−‖*p* − *q*‖^2^/*σ*_*r*_^2^) and exp(−‖*P*_*p*_ − *Q*_*q*_‖^2^/*σ*_*r*_^2^) defining the contribution of pixel intensity ranges. If *Q* and *P* are equal, (2) is shortened as a single image smoothing procedure.

The article "Atom Search Optimization with the Deep Transfer Learning-Driven Esophageal Cancer Classification Model" was retracted in 2023. Reasons: signs of a paper mill; suspected computer-generated content; unreliable results or conclusions; concerns about the data.

### 3.2. Deep Transfer Learning Model

Once the medical image is preprocessed, the next phase is developing a useful feature vector set utilizing ResNet 101. A CNN [20] is generally comprised of alternative max‐pooling and convolutional layers (represented as *P* and *C* layers) for hierarchically extracting features from the original input, followed by a fully connected (FC) layer to perform classification. Considering a CNN with *L* layers, we represented the output state of *l*-*th* layer as *H*^*l*^, whereas *l* ∈ {1,…, *L*}, with *H*^0^ representing the input dataset. There are two parts of the training parameter in all the layers that are weight matrix *W*_*l*_ which connect the *l*-*th* layers and the preceding layers using *H*^*l*−1^, and the bias vector refers to *b*_*l*_. The input dataset is generally interconnected with *C* layer. For *C* layer, a 2D convolutional function is implemented initially with convolution kernel *W*_*l*_. Next, the bias *b*_*l*_ is included in the resulting feature map where a pointwise nonlinear activation function *g*(∙) is widely implemented. At last, a max‐pooling layer is generally followed to choose the dominant feature over the nonoverlapping square window for all the feature maps.

(3) $$\begin{array}{c} H^{l}=pool\left(g\left(H^{l-1}*W_{l}+b_{l}\right)\right)\text{.} \end{array}$$

In (3), the convolution operation is denoted by the symbol *∗* and pool indicates the max‐pooling function. *C* and *P* layers are stacked one after another to form the feature extraction hierarchically. Next, the resulting feature is integrated with a 1D feature vector with the FC layer. Initially, the FC layer processes the input using nonlinear conversion using weight *W*_*l*_ and bias *b*_*l*_ as follows:

(4) $$\begin{array}{c} H^{l}=g\left(H^{l-1}*W_{l}+b_{l}\right)\text{.} \end{array}$$

Many nonlinear activation functions were introduced. Now, we selected the sigmoid activation for its higher efficiency and capability:

(5) $$\begin{array}{c} g\left(x\right)={\left(1|+\right.}^{\left.\exp^{\left(-x\right)}\right)-1}\text{.} \end{array}$$

The final classification layer is generally a SoftMax layer, with neuron count equalizing the class count to be categorized. Then, utilize an LR layer with a single neuron to perform dual classification, i.e., analogous to the FC layer. The weight {*W*_1_, ⋯, *W*_*L*_} and the bias {*b*_1_, ⋯, *b*_*L*_} compose the model parameter that is jointly and iteratively augmented by maximizing the classification performance over the training set.  Figure 2 illustrates the structure of residual learning.

The article "Atom Search Optimization with the Deep Transfer Learning-Driven Esophageal Cancer Classification Model" was retracted in 2023. Reasons: signs of a paper mill; suspected computer-generated content; unreliable results or conclusions; concerns about the data.

ResNet101 is a CNN that comprises fifty layers; it can be deeper than VGG-16. Because a global average pool was utilized rather than an FC layer, the model size was significantly smaller and decreases the ResNet101 size by 102 MB [21]. The ResNet is a distinctive part of residual block learning which implies that all the layers must feed into the following layer around 2-3 hops away. The substructure is comprised of the following:

- The convolutional layer has KS (KS) of 7 × 7 and 64 filters. It is followed by a max pooling layer with a stride size of 2.
- Next, a convolution layer has KS of 1∗1 and 64 filters; after that, the next convolution layers have a KS of 3∗3 and 64 filters. Later, we have other convolution layers with a KS of 1∗1 and 256 filters. These three layers are replicated 3 times and 9 layers are attained during this phase.
- Then, three convolution layers are as follows: the initial one with a KS of 1∗1 and 128 filters, the next one with a KS of 3∗3and 128 filters, and the last one with a KS of 1∗1 and 512 filters. This layer is replicated 4 times to provide 12 layers during this phase.
- Later, we have a convolution layer with KSs of 1∗1 and 256 filters, with KSs of 3∗3 and 2 56 filters, with a KS of 1 ∗ 1 and 1024 filters. It can be replicated 6 times to provide a total of 18 layers.
- After that, we have a convolution layer with KS of 1∗1 and512 filters, with a KS of 1 ∗ 1 and 512 filters, with a kernel of 3 ∗ 3 and 2048 filters. It can be replicated 3 times to provide a total of 9 layers.
- Lastly, an average pooling can be used and FC layer is used to complete them (1000 nodes) and a SoftMax function to provide 1 layer as the last phase.

### 3.3. EC Classification Model

In this study, the feature vectors are passed into the ELM model to identify EC [22]. ELM is an alternate name for one or more hidden layer feedforward neural networks (FFNN). ELM is utilized for solving feature engineering, classification, clustering, and regression problems. This learning approach includes the output layer, input layer, and one or multiple hidden layers. In the conventional neural network, the task of fine-tuning the hidden and input layers is time‐consuming and computationally expensive since it needs numerous rounds to converge. The performance of ELM is similar to SVM or other ML classifier models. ELM has a greater capacity for better performing in very sophisticated datasets. *N* input instance (*z*_*i*_, *y*_*i*_) are presented, in which *z*_*i*_=[*x*_*i*1_, *x*_*i*2_, ⋯⋯,*x*_*in*_]^*T*^ indicates the *i*-*th* samples with *n* discrete features and *y*_*i*_=[*y*_*i*1_, *y*_*i*2_, ⋯⋯,*y*_*im*_]^*T*^ defines the original label of *x*_*i*_ with conventional SLFN using *K* hidden neurons that are determined:

(6) $$\begin{array}{c} \overset{K}{\underset{m=1}{\sum }}\beta_{i}h\left(w_{m}.x_{i}+c_{m}\right)=\alpha_{i},i=1,\cdots \cdots \cdots ,N\text{.} \end{array}$$

In (6), *β*_*i*_=[*β*_*i*1_, *β*_*i*2_, ⋯⋯,*β*_*im*_]^*T*^ illustrates the weight vector with the connection of *i*-*th* hidden layers and the output node, *w*_*m*_=[*w*_*m*1_, *w*_*m*2_, ⋯⋯,*w*_*mn*_]^*T*^ refers to the selected weight vector and represents *i*-*th* hidden layers with the input node, and *c*_*m*_ denotes the threshold of *i*-*th* hidden layers. *α*_*k*_=[*α*_*k*1_, *α*_*k*2_, ⋯⋯,*α*_*km*_]^*T*^ refers to the *k*-*th* output neurons. *h* stands for the activation function and SLFN is applied to *M* hidden neuron and activation function approaches *N* trainable instance with zero errors. Many other technologies were used to classify and detect intrusions of wireless and wired environments.  Figure 3 depicts the framework of ELM.

The article "Atom Search Optimization with the Deep Transfer Learning-Driven Esophageal Cancer Classification Model" was retracted in 2023. Reasons: signs of a paper mill; suspected computer-generated content; unreliable results or conclusions; concerns about the data.

### 3.4. Parameter Optimization

The ASO algorithm has been utilized to improve the EC classification performance of the ASODTL-ECC model [23]. The presented ASO algorithm is based on molecular dynamics. In the searching space, the position of each atom defines its calculation and the clarification based on mass and provides a better solution. ASO continues the streamlining procedure by making a considerable amount of arrangements randomly. For each loop, the particle changes its locations and speeds, along with the location of the best atom. Moreover, particle acceleration can be classified into two segments. The initial one is the collaboration force that can be determined as an L‐j potential is generally the fascination from various particles and vector sum of aversion. It is confronted with the potential of particle and bond length in addition to the finest particle is weighted position difference because of the required energy. The computation satisfies the broken model, and it is logically implemented. The best atom fitness and location are reverted, and the global optimal is predictable. The fitness function is utilized for determining the maximum benefit parameter as per the objective function. The fitness function can be described in the following expression:

(7) $$\begin{array}{c} M^{a}\left(T\right)=e\frac{-Fit^{a}\left(T\right)-Fit^{a}\left(T\right)}{Fit_{worst}^{a}\left(T\right)}\text{.} \end{array}$$

In order to evaluate the simple level of the fitness function, the mass of an atom is calculated by

(8) $$\begin{array}{c} m^{a}\left(T\right)=\frac{M^{a}\left(T\right)}{\Sigma_{n=1}^{N}M^{b}\left(T\right)}\text{.} \end{array}$$

In (8), *Fit*_best_^*a*^(*T*) stands for the minimal fitness values and *Fit*_worst_^*a*^(*T*) is defined by the maximal fitness value in *t*-*th* iterations. *Fit*^*a*^(*T*) is referred to as the fitness function of *t*-*th* iteration of *i*-*th* atoms. The *C* neighbor is evaluated according to the following expression, in which *a*,*b* terms are represented as atoms.

(9) $$\begin{array}{c} C\left(T\right)=N-\left(N-2\right)\times \sqrt{\frac{T}{t}}\text{.} \end{array}$$

In the detection method of the ASA approach, all the atoms need a considerable amount of atoms with the fitness parameter of the *k* neighbor. Atom was predictable to relate through as specific atom with fitness parameter since *C* neighbor boosts exploitation in the last phase of iterations. Equation (9) is utilized for calculating the *C* neighbors: *T* stands for maximal iterations, *N* for size of population, and *t* for dimension in time. The property of acceleration and atomic contact force is computed, and various mechanisms of weight employed to the *i*-*th* atoms from the atom of force are formulated:

(10) $$\begin{array}{c} F_{a}^{D}\left(T\right)=\overset{n}{\underset{bebest}{\sum }}ran\;dom_{b}f_{ab}^{D}\left(T\right)\text{.} \end{array}$$

In (10), random refers to a random integer within [0,1]; *f* represents fitness function. The acceleration is computed by the following expression:

(11) $$\begin{array}{c} G_{a}^{D}\left(T\right)=\alpha \left(T\right)\left(X_{best}^{D}\left(T\right)-X_{a}^{D}\left(T\right)\right)\text{.} \end{array}$$

The Lagrangian multiplier is determined by

(12) $$\begin{array}{c} \alpha \left(T\right)=\beta e^{-20T/t}\text{.} \end{array}$$

In (12), *β* is determined by the multiplier weight. In the updating procedure, the velocity and position of *i*-*th* atom at the condition of (*t*+1)*th* iterations are represented as follows:

(13) $$\begin{array}{c} \begin{array}{c} V_{a}^{D}\left(t+1\right)=rand_{a}^{D}V_{a}^{D}\left(T\right)+A_{a}^{D}\left(t\right)\\ X_{a}^{D}\left(t+1\right)=X_{a}^{D}\left(t\right)+V_{a}^{D}\left(t+1\right) \end{array}\text{.} \end{array}$$

The best approach for minimizing power quality problems and accomplishing the exercise function is carefully chosen after the upgrading procedure. The last condition needs to be verified beforehand by utilizing the optimum solution, where the maximal iteration is attained and constraint is calculated. The pseudocode of ASO is provided in Algorithm 1.

The article "Atom Search Optimization with the Deep Transfer Learning-Driven Esophageal Cancer Classification Model" was retracted in 2023. Reasons: signs of a paper mill; suspected computer-generated content; unreliable results or conclusions; concerns about the data.

The ASO system extracts a fitness function for achieving enhanced classification act. It fixes a positive integer for representing the superior outcomes of the candidate solutions. In this article, the reduction of the classification fault rate is assumed as the fitness function, as provided in the following equation:

(14) $$\begin{array}{c} fitness\left(x_{i}\right)=ClassifierErrorRate\left(x_{i}\right)\frac{number\;of\;misclassifie\;d\;samples}{Total\;number\;of\;samples}*100\text{.} \end{array}$$

## 4. Results and Discussion

The experimental validation of the ASODTL-ECC model is tested using a set of images, as given in Table 1. The results are inspected under three subdatasets, namely, entire dataset, 70% of training (TR) data, and 30% of testing (TS) data.  Figure 4 showcases the sample images.

Figure 5 displays the confusion matrices created by the ASODTL-ECC model on the applied dataset. With the entire dataset, the ASODTL-ECC model has identified 249, 238, and 248 samples under classes 0, 1, and 2, respectively. Meanwhile, with 70% of the TR dataset, the ASODTL-ECC approach has identified 163, 174, and 174 samples under classes 0, 1, and 2, respectively. Eventually, with 30% of the TS dataset, the ASODTL-ECC algorithm has identified 86, 64, and 74 samples under classes 0, 1, and 2, respectively.

Table 2 illustrates a detailed EC classification result of the ASODTL-ECC model on distinct sizes of data.  Figure 6 portrays a comprehensive EC classification performance of the ASODTL-ECC model on the entire data. The figure indicated that the ASODTL-ECC model has recognized all class labels. For instance, the ASODTL-ECC model has recognized class 0 samples with *accu*_*y*_, *sens*_*y*_, *spec*_*y*_, *F*_score_, MCC, and *J*_in de x_ of 99.93%, 99.60%, 99.20%, 99.01%, 98.51%, and 98.03% respectively. Along with that, the ASODTL-ECC system has recognized class 1 samples with *accu*_*y*_, *sens*_*y*_, *spec*_*y*_, *F*_score_, MCC, and *J*_in de x_ of 98.27%, 95.20%, 99.80%, 97.34%, 96.11%, and 94.82%, respectively. Therefore, the ASODTL-ECC algorithm has recognized class 2 samples with *accu*_*y*_, *sens*_*y*_, *spec*_*y*_, *F*_score_, MCC, and *J*_in de x_ of 98.40%, 99.20%, 98%, 97.64%, 96.46%, and 95.38%, respectively.

The article "Atom Search Optimization with the Deep Transfer Learning-Driven Esophageal Cancer Classification Model" was retracted in 2023. Reasons: signs of a paper mill; suspected computer-generated content; unreliable results or conclusions; concerns about the data.

Figure 7 demonstrates a comprehensive EC classification performance of the ASODTL-ECC technique on 70% of TR data. The figure exposed that the ASODTL-ECC approach has recognized all class labels. For instance, the ASODTL-ECC technique has recognized class 0 samples with *accu*_*y*_, *sens*_*y*_, *spec*_*y*_, *F*_score_, MCC, and *J*_in de x_ of 99.05%, 99.39%, 98.89%, 98.49%, 97.80%, and 97.02%, respectively. Besides, the ASODTL-ECC model has recognized class 1 samples with *accu*_*y*_, *sens*_*y*_, *spec*_*y*_, *F*_score_, MCC, and *J*_in de x_ of 97.71%, 94.05%, 99.71%, 96.67%, 95.01%, and 93.55%, respectively. Likewise, the ASODTL-ECC approach has recognized class 2 samples with *accu*_*y*_, *sens*_*y*_, *spec*_*y*_, *F*_score_, MCC, and *J*_in de x_ of 97.90%, 98.86%, 97.42%, 96.94%, 94.39%, and 94.05%, respectively.

Figure 8 illustrates a comprehensive EC classification performance of the ASODTL-ECC approach on 30% of TS data. The figure represented that the ASODTL-ECC technique has recognized all class labels. For instance, the ASODTL-ECC model has recognized class 0 samples with *accu*_*y*_, *sens*_*y*_, *spec*_*y*_, *F*_score_, MCC, and *J*_in de x_ of 100%, 100%, 100%, 100%, 100%, and 100%, respectively. Then, the ASODTL-ECC algorithm has recognized class 1 samples with *accu*_*y*_, *sens*_*y*_, *spec*_*y*_, *F*_score_, MCC, and *J*_in de x_ of 99.56%, 98.46%, 100%, 99.22%, 98.92%, and 98.46%, respectively. Eventually, the ASODTL-ECC methodology has recognized class 2 samples with *accu*_*y*_, *sens*_*y*_, *spec*_*y*_, *F*_score_, MCC, and *J*_in de x_ of 99.56%, 100%, 99.34%, 99.33%, 99%, and 98.67%, respectively.

The training accuracy (TA) and validation accuracy (VA) attained by the ICSOA-DLPEC methodology on the test dataset are demonstrated in Figure 9. The experimental outcome implied that the ICSOA-DLPEC technique has gained maximal values of TA and VA. Specifically, the VA seemed to be higher than TA.

The training loss (TL) and validation loss (VL) achieved by the ICSOA-DLPEC system on the test dataset are established in Figure 10. The experimental outcome inferred that the ICSOA-DLPEC approach had achieved the least values of TL and VL. Specifically, the VL seemed to be lower than TL.

A brief precision-recall examination of the ASODTL-ECC approach on the test dataset is represented in Figure 11. By observing the figure, it can be noticed that the ASODTL-ECC model has accomplished maximal precision-recall performance under all classes.

A detailed ROC investigation of the ASODTL-ECC methodology on the test dataset is depicted in Figure 12. The outcomes indicated that the ASODTL-ECC model has displayed its ability to categorize three different classes 0–2 on the test dataset.

The article "Atom Search Optimization with the Deep Transfer Learning-Driven Esophageal Cancer Classification Model" was retracted in 2023. Reasons: signs of a paper mill; suspected computer-generated content; unreliable results or conclusions; concerns about the data.

The comparative investigation of the results offered by the ASODTL-ECC model is provided in Table 3 [24, 25].  Figure 13 offers a clear comparison analysis of the ASODTL-ECC model with recent techniques with respect to *sens*_*y*_, *spec*_*y*_, and *F*_score_. The figure outperformed that the EfficientNet-B0, RegNetY-400 MF, DenseNet201, and GoogLeNet algorithms have exhibited lesser values of *sens*_*y*_, *spec*_*y*_, and *F*_score_. Besides, VGG-16 and ResNet18 algorithms have displayed moderately closer values of *sens*_*y*_, *spec*_*y*_, and *F*_score_. Eventually, the ResNet50 model has accomplished reasonably *sens*_*y*_, *spec*_*y*_, and *F*_score_ of 97.06% 93.62%, and 94.77%, respectively, the ASODTL-ECC methodology has obtained maximal *sens*_*y*_, *spec*_*y*_, and *F*_score_ of 99.49%, 99.78%, and 99.52%, respectively.

Figure 14 provides a clear comparison study of the ASODTL-ECC model with recent models in terms of *accu*_*y*_. The figure indicated that the EfficientNet-B0, RegNetY-400 MF, DenseNet201, and GoogLeNet models have shown lower values of *accu*_*y*_. At the same time, VGG-16 and ResNet18 models have demonstrated moderately closer values of *accu*_*y*_. Though the ResNet50 model has accomplished reasonable *accu*_*y*_ of 97.06%, the ASODTL-ECC model has obtained a maximum *accu*_*y*_ of 99.49%.

From the detailed results and discussion, it is apparent that the ASODTL-ECC model has accomplished effectual outcomes on EC classification.

## 5. Conclusion

In this study, a novel ASODTL-ECC model has been developed to investigate the medical images for the existence of EC in a timely and accurate manner. The presented ASODTL-ECC model encompasses various subprocesses, namely, GF-based noise elimination, ResNet-based feature extraction, ELM classification, and ASO-based parameter tuning. The use of the ASO algorithm assists in improving the identification of the presence of EC. The performance of the ASODTL-ECC model is assessed and compared with existing models under several medical images. The experimental results pointed out the improved performance of the ASODTL-ECC model over recent approaches. Thus, the ASODTL-ECC model can be exploited for effectual EC detection and classification process. In the future, an ensemble of DTL models can be applied to improve the detection efficiency of the ASODTL-ECC model. In addition, the computational complexity of the proposed model can be studied in our future work.

## Figures and Tables

**Figure 1:** Block diagram of the ASODTL-ECC technique.

The article "Atom Search Optimization with the Deep Transfer Learning-Driven Esophageal Cancer Classification Model" was retracted in 2023. Reasons: signs of a paper mill; suspected computer-generated content; unreliable results or conclusions; concerns about the data.

**Figure 2:** Structure of residual learning.

**Figure 3:** Framework of the ELM method.

**Figure 4:** Sample images.

**Figure 5:** Confusion matrices of the ASODTL-ECC technique: (a) entire dataset, (b) 70% of TD data, and (c) 30% of TS data.

**Figure 6:** Result analysis of the ASODTL-ECC technique under entire dataset.

**Figure 7:** Result analysis of the ASODTL-ECC technique under 70% of TR data.

**Figure 8:** Result analysis of the ASODTL-ECC technique under 30% of TS dataset.

**Figure 9:** TA and VA analysis of the ASODTL-ECC technique.

**Figure 10:** TL and VL analysis of the ASODTL-ECC technique.

**Figure 11:** Precision-recall curve analysis of the ASODTL-ECC technique.

**Figure 12:** ROC curve analysis of the ASODTL-ECC technique.

**Figure 13:** Comparative analysis of the ASODTL-ECC technique with recent algorithms.

**Figure 14:** *Accu*_*y*_ analysis of the ASODTL-ECC technique with recent algorithms.

**Algorithm 1:** Pseudocode of ASO algorithm.

**Table 1:** Dataset details.

Label	Class name	No. of images
Class 0	Normal	250
Class 1	Esophagitis	250
Class 2	Esophagus cancer	250
Total number of images		**750**

**Table 2:** Result analysis of the ASODTL-ECC technique with various measures.

Label	Accuracy	Sensitivity	Specificity	F-score	MCC	Jaccard index
Entire dataset						
Class 0	99.33	99.60	99.20	99.01	98.51	98.03
Class 1	98.27	95.20	99.80	97.34	96.11	94.82
Class 2	98.40	99.20	98.00	97.64	96.46	95.38
**Average**	**98.67**	**98.00**	**99.00**	**98.00**	**97.02**	**96.08**

Training phase (70%)						
Class 0	99.05	99.39	98.89	98.49	97.80	97.02
Class 1	97.71	94.05	99.71	96.67	95.01	93.55
Class 2	97.90	98.86	97.42	96.94	95.39	94.05
**Average**	**98.22**	**97.44**	**98.67**	**97.36**	**96.07**	**94.88**

Testing phase (30%)						
Class 0	100.00	100.00	100.00	100.00	100.00	100.00
Class 1	99.56	98.46	100.00	99.22	98.92	98.46
Class 2	99.56	100.00	99.34	99.33	99.00	98.67
**Average**	**99.70**	**99.49**	**99.78**	**99.52**	**99.31**	**99.04**

**Table 3:** Comparative analysis of the ASODTL-ECC technique with existing algorithms.

Methods	Sensitivity	Specificity	Accuracy	F-score
VGG-16	96.40	98.06	94.42	90.35
ResNet18	96.31	95.78	92.73	91.03
ResNet50	97.06	93.62	94.77	96.20
EfficientNet-B0	92.14	97.75	95.58	96.39
RegNetY-400 MF	92.15	90.91	92.83	95.49
DenseNet201	92.68	92.43	92.97	96.18
GoogLeNet	92.09	91.77	91.89	93.88
ASODTL-ECC	99.49	99.78	99.7	99.52

## Data Availability

Data sharing is not applicable to this article as no datasets were generated during the current study.
